The article "CT-Based Risk Factors for Mortality of Patients With COVID-19 Pneumonia in Wuhan, China: A Retrospective Study" was retracted in 2023. Reasons: unreliable results or conclusions; lack of ethics approval or compliance; concerns about the data; concerns about the results or conclusions.

# CT-Based Risk Factors for Mortality of Patients With COVID-19 Pneumonia in Wuhan, China: A Retrospective Study

**DOI:** 10.3389/fradi.2021.661237

**Published:** 2021-07-01

**Authors:** Xiang Li, Nannan Li, Zhen Chen, Ling Ye, Ling Zhang, Dakai Jin, Liangxin Gao, Xinhui Liu, Bolin Lai, Jiawen Yao, Dazhou Guo, Hua Zhang, Le Lu, Jing Xiao, Lingyun Huang, Fen Ai, Xiang Wang

**Affiliations:** ^1^The Central Hospital of Wuhan Affiliated to Tongji Medical College of Huazhong University of Science and Technology, Wuhan, China; ^2^Intelligent Vision Technology Department, Ping An Technology, Shenzhen, China; ^3^PAII Inc., Bethesda, MD, United States; ^4^Linking Med, Beijing, China

**Keywords:** COVID-19, risk factor, mortality, computed tomography, artificial intelligence system

## Abstract

**Purpose:** Computed tomography (CT) characteristics associated with critical outcomes of patients with coronavirus disease 2019 (COVID-19) have been reported. However, CT risk factors for mortality have not been directly reported. We aim to determine the CT-based quantitative predictors for COVID-19 mortality.

**Methods:** In this retrospective study, laboratory-confirmed COVID-19 patients at Wuhan Central Hospital between December 9, 2019, and March 19, 2020, were included. A novel prognostic biomarker, V-HU score, depicting the volume (V) of total pneumonia infection and the average Hounsfield unit (HU) of consolidation areas was automatically quantified from CT by an artificial intelligence (AI) system. Cox proportional hazards models were used to investigate risk factors for mortality.

**Results:** The study included 238 patients (women 136/238, 57%; median age, 65 years, IQR 51–74 years), 126 of whom were survivors. The V-HU score was an independent predictor (hazard ratio [HR] 2.78, 95% confidence interval [CI] 1.50–5.17; *p* = 0.001) after adjusting for several COVID-19 prognostic indicators significant in univariable analysis. The prognostic performance of the model containing clinical and outpatient laboratory factors was improved by integrating the V-HU score (c-index: 0.695 vs. 0.728; *p* < 0.001). Older patients (age ≥ 65 years; HR 3.56, 95% CI 1.64–7.71; *p* < 0.001) and younger patients (age < 65 years; HR 4.60, 95% CI 1.92–10.99; *p* < 0.001) could be further risk-stratified by the V-HU score.

**Conclusions:** A combination of an increased volume of total pneumonia infection and high HU value of consolidation areas showed a strong correlation to COVID-19 mortality, as determined by AI quantified CT.

## Introduction

The highly contagious coronavirus disease 2019 (COVID-19), broke up in 2019, has spread worldwide, posing a great threat to public health (1). As of the 29th of October, 2020, global coronavirus deaths have surpassed one million. As the confirmed cases and deaths dramatically increase, intensive-care units are nearly overwhelmed, and medical resources are of a dire shortage. In facing such a pandemic, finding out the risk factors associated with death and thus taking timely care toward those high-risk patients has the potential to reduce the mortality rate.

Currently, albeit the reverse-transcriptase-polymerase-chain-reaction test is used as the standard reference for diagnosing COVID-19, it often suffers from false negatives and longer turnaround times (2). In the context of typical clinical presentation and exposure to other individuals with COVID-19, it may result in quarantine omission, acceleration of COVID-19 spread, consequently worsening the pandemic. In many countries of Europe and Asia, CT imaging-based examination protocol stands out and becomes a complementary tool for the COVID-19 diagnosis with merits of high sensitivity to viral infection, easy access for patients, and quick acquisition of imaging (3, 4).

Following the COVID-19 pandemic spreading, research activities on COVID-19 have become very active. Epidemiological, clinical, laboratory and radiologic characteristics of COVID-19 are summarized in previous studies (5–9). Clinical and laboratory risk factors for critical illness or death are also analyzed (6, 10–13), where age is a well-recognized significant predictor in all studies, with additional clinical and laboratory factors or indices composed of multiple factors, such as d-dimer and SOFA score (10), MuLBSTA score (6), CD3+CD8+ T-cells and cardiac troponin levels (12), and deep-survival score involving neutrophil count and lactate dehydrogenase (13). On the other hand, several recent studies also demonstrate that chest CT imaging has great prognostic value for COVID-19 (14–16). The volumes or volume ratios of lung infections, e.g., total lesion, or ground-glass opacity (GGO), are shown to be predictors of substantial outcomes (ICU admission and death) (14, 15). Here, the direct correlation of quantitative CT features with the COVID-19 mortality in our patient cohort was explored.

In this study, we aim to investigate the CT based radiologic risk factors associated with COVID-19 mortality. The radiologic factors were automatically computed using an AI-based pulmonary imaging analysis system and validated with demographic, clinical, and laboratory risk factors.

## Materials and Methods

### Study Design and Participants

In this retrospective study, patients diagnosed as COVID-19 in line with WHO interim guidance at Wuhan Central Hospital from December 9, 2019, to March 19, 2020, were enrolled (17). Our inclusion criteria were: (i) reverse-transcriptase-polymerase-chain-reaction confirmed COVID-19; (ii) chest CT scanning at diagnosis time and revealing a typical ground glass shadow in lungs; (iii) with the final outcome (i.e., survival or dead) recorded. Ultimately, 238 patients with 238 CTs were enrolled. For the prognostic analysis, we defined the first CT examination time as the start point. CT imaging protocol was described in Supplementary Methods. The study was approved by the Research Ethics Commission of Wuhan Central Hospital, and written informed consent was waived by the Ethics Commission for the emergence of infectious diseases.

### Data Collection

We reviewed the clinical electronic medical records, nursing records, laboratory findings, and radiological examinations for all patients with COVID-19. Epidemiological, demographic, clinical, laboratory, and outcome data were extracted using a standardized data collection form.

### CT Image Analysis

The whole lung field, pneumonia infection regions, and pleural effusion regions were first segmented using a fully-automated AI-based pulmonary imaging analysis system (Supplementary Methods) (18). Then according to the Hounsfield unit (HU) values, infection regions were further divided into GGO and consolidation by setting threshold values (19). Areas with HU values > −200 were regarded as consolidation, and those between −700 and −200 were regarded as GGO. Segmentation network architectures were illustrated in the Supplementary Figures 3–5.

CT imaging features were computed based on the size and attenuation of infection regions. Specifically, we calculated infection volumes, volume ratios (%) of the infection regions to the whole lung field, and average HU values of the total pneumonia infection, GGO, consolidation, and pleural effusion. Using these features, we further calculated a discrete V-HU score, as the proposed imaging biomarker, taking both the volume of total pneumonia infection (V) and the average HU value of the consolidation region (HU) into account. V-HU was mainly categorized into three groups according to different extent of pulmonary damage with different values of V and HU. Specifically, the V-HU score was set to “0” (referring to the low-risk group) if both the V and the HU were less than the corresponding median values in study participants. Similarly, the V-HU score was set to “2” (referring to the high-risk group) only if both the V and the HU were larger than the corresponding median values in study participants. We set the V-HU score to “1” (referring to the intermediate-risk group) for other conditions.

### Evaluation of Our AI System on Lesion Segmentation Tasks

To evaluate the performance of our AI semantic *segmentation* framework, an internal validation set of 121 slices from 30 COVID-19 patients were manually annotated at the pixel level into three classes, including ground-glass opacity (GGO), consolidation, and pleural effusion regions. Two junior radiologists with over-5-year clinical experience were employed to delineate the total pneumonia infection, pleural effusion and lung field regions. Then three senior radiologists with over-15-year clinical experience were asked to check the annotations. Ultimately, ground truth can be acquired based on the consistency among the senior radiologists. We evaluated the performance of our automatic segmentation network using Dice Coefficient (Dice) as a measure of overlap between predicted segmentation labels and ground truth segmentation labels. A coefficient of 1 means that the predicted segmentation labels and ground truth segmentation labels are perfectly matched, while 0 means there is no overlap between them.

### Statistical Analysis

Continuous variables were expressed as median with interquartile range (IQR), and categorical variables were presented as frequency with percentages (%). Differences between survivors and non-survivors were evaluated by Mann-Whitney U test for continuous variables and Chi-square test or Fisher's exact test for categorical variables as appropriate. A two-sided α of < 0.05 was considered statistically significant.

Univariable and multivariable Cox proportional-hazards models were used to examine the association between the risk factors and patient outcomes. In-hospital death was assessed with four multivariable models under four different clinical circumstances: model 1 (simulating inpatients with CT scans) included all the seven most significant factors selected from univariable Cox model analysis containing demographic, clinical, inpatient, outpatient laboratory parameters, and our radiologic marker; model 2 (simulating outpatients without CT scans) included demographic, clinical, and outpatient laboratory factors; model 3 (simulating inpatients without CT scans) included demographic, clinical, both outpatient and inpatient laboratory factors; model 4 (simulating outpatients with CT scans) included demographic, clinical, outpatient laboratory and our radiologic marker. The selection of model covariates was detailed below.

For the missing laboratory parameters for which the overall deficiency rate was no more than 25%, we adopted a multivariable imputation approach, i.e., *aregImpute* (20). By fitting flexible additive imputation models from non-missing data, target variables can be predicted through bootstrap resamples from a full Bayesian predictive distribution. See Supplementary Methods for detailed missing laboratory parameters. The data imputation process was carried out using “*Hmisc*” (v4.4.0) of R software.

Continuous variables were binarized by their corresponding median values as cutoffs. Significant variables (*p* < 0.05) in univariable analysis were considered as candidate variables for multivariable analysis. Considering the limited number of events, up to seven variables were chosen for multivariable analysis to avoid overfitting in the models. If there were several strongly correlated variables, only the most significant variable was included in the multivariable analysis. The correlation between any two variables in the univariable analysis was illustrated in the Supplementary Figure 6. White blood cell count (*p* = 6.06*e*^−6^) was not included in the model because of a strong correlation with the neutrophil count (*p* = 1.05*e*^−6^). For the correlated radiologic variables, only the most significant one, the V-HU score, was used in the multivariable analysis, since it considered both the volume and attenuation of the pneumonia infection. Mortalities in the V-HU-defined subgroups were described using Kaplan-Meier analysis, and the log-rank test was used to assess whether the marker predicted mortality. All model-based results were presented with 95% CI.

All statistical analyses were conducted using Python 3.6 libraries unless otherwise indicated. We used pandas (0.24.2) for calculating IQR and correlation matrices. Chi-square test and Mann-Whitney *U*-test were done with scipy (1.3.0). Cox proportional-hazards models and Kaplan-Meier curves were done with lifelines (0.24.6).

## Results

The study initially collected 244 patients who met abovementioned inclusion criteria. Since large quantities of mildly ill patients did not come for further consultation, they were not included in this study owing to the absence of follow-up records. Among the collected patients, six patients lacking laboratory parameters were excluded. Ultimately, the study sample consisted of 238 COVID-19 patients (Figure 1). Demographic, clinical, and laboratory characteristics (obtained from outpatient and inpatient examinations) are reported in Table 1. The median age of the patients was 65 years (IQR, 51–74). Non-survivors were older than survivors (median 70, IQR 63–80 vs. median 57, IQR 37–68; *p* < 0.001). Non-survivors had a higher percentage of patients aged >75 years than survivors (40/112, 36% vs. 13/126, 10%). Women made up 57% (136/238) of all patients but accounted for 69% (77/112) of the non-survivors. Fever was a common symptom (171/236, 72%) in all patients with temperature records. Non-survivors had a higher prevalence of cerebrovascular disease (20/112, 18% vs. 3/126, 2.4%), hypertension (49/112, 44% vs. 38/126, 30%), cardiovascular disease (25/112, 22% vs. 17/126, 13%), diabetes (25/112, 22% vs. 21/126, 17%), and other comorbidity (32/112, 29% vs. 33/126, 26%) than survivors. For the laboratory parameters, a higher percentage of non-survivors than survivors presented with elevated levels of c-reactive protein, white blood cell count, neutrophil count, d-dimer, and lactic dehydrogenase.

**Figure 1:** Diagram showing the patient selection process. COVID-19, Coronavirus Disease 2019; CT, computed tomography.

**Table 1:** Demographic, clinical and laboratory characteristics of 238 COVID-19 patients.

	**ALL (*n* = 238)**	**Survivor (*n* = 126)**	**Non-survivor (*n* = 112)**	***p*-value**
**Demographics and clinical characteristics**				
Age (years)	65 (51–74)	57 (37–68)	70 (63–80)	< 0.001
< =40	43/238 (18%)	42/126 (33%)	1/112 (89%)	< 0.001
40–65	83/238 (35%)	47/126 (37%)	36/112 (32%)	
65–75	59/238 (25%)	24/126 (19%)	35/112 (31%)	
>75	53/238 (22%)	13/126 (10%)	40/112 (36%)	
Sex				
Men	102/238 (43%)	67/126 (53%)	35/112 (31%)	< 0.001
Women	136/238 (57%)	59/126 (47%)	77/112 (69%)	
Temperature	37.9 (37.2–38.5)	38.0 (37.4–38.6)	37.8 (37.1–38.2)	0.03
Fever (≥37.3)	171/236 (72%)	97/126 (77%)	74/110 (67%)	0.096
Comorbidity	150/238 (63%)	68/126 (54%)	82/112 (73%)	0.002
Cardiovascular disease	42/238 (18%)	17/126 (13%)	25/112 (22%)	0.08
Hypertension	87/238 (37%)	38/126 (30%)	49/112 (44%)	0.030
Cerebrovascular disease	23/238 (10%)	3/126 (2.4%)	20/112 (18%)	< 0.001
Diabetes	46/238 (19%)	21/126 (17%)	25/112 (22%)	0.27
Others	65/238 (27%)	33/126 (26%)	32/112 (29%)	0.68
**Outpatient laboratory parameters**				
White blood cell count (× 10^9^per L)	5.9 (4.3–8.02)	5.1 (3.9–6.7)	7.01 (5.2–9.2)	< 0.001
< =4	49/231 (21%)	33/122 (27%)	16/109 (15%)	< 0.001
4–10	151/231 (65%)	82/122 (67%)	69/109 (63%)	
>10	31/231 (13%)	7/122 (5.7%)	24/109 (22%)	
Neutrophil count (× 10^9^per L)	4.5 (2.97–7.9)	3.6 (2.6–5.9)	6.4 (3.9–9.3)	< 0.001
>3.6	145/229 (63%)	60/121 (50%)	85/108 (79%)	< 0.001
lymphocyte count (× 10^9^per L)	0.8 (0.5–1.1)	0.9 (0.6–1.2)	0.7 (0.5–0.95)	< 0.001
< =0.8	118/231 (51%)	55/122 (45%)	63/109 (58%)	0.05
C-Reactive Protein (mg/L)	3.8 (1.5–7.8)	2.3 (0.6–6.1)	5.4 (3.1–10.7)	< 0.001
>1	174/218 (80%)	80/118 (68%)	94/100 (94%)	< 0.001
**Inpatient laboratory parameters**				
Blood Oxygen	60.0 (49.0–80.0)	68.5 (56.5–87.0)	56.0 (45.5–73.5)	< 0.001
< =80%	136/181 (75%)	57/86 (66%)	79/95 (83%)	0.01
D-dimer (μg/L)	2.2 (0.7–7.7)	1.1 (0.6–4.7)	4.7 (1.4–9.3)	< 0.001
< =0.5	23/182 (13%)	20/95 (21%)	3/87 (3.0%)	< 0.001
0.5–1	35/182 (19%)	25/95 (26%)	10/87 (11%)	
>1	124/182 (68%)	50/95 (53%)	74/87 (85%)	
lactic dehydrogenase (U/L)	316.0 (214.0–450.0)	244.0 (187.0–350.0)	406.5 (263.8–576.8)	< 0.001
>245	113/177 (64%)	44/89 (49%)	69/88 (78%)	< 0.001

*Data are median (IQR), n (%), or n/N (%). p-values were calculated by Mann-Whitney U-test, Chi-square test, or Fisher's exact test, as appropriate*.

The whole lung field and pneumonia infected regions from CT scans were automatically segmented and quantified using our pulmonary AI analysis system. The mean 2D Dice score and standard deviation of internal validation set over each segmentation task were summarized in Table 2. Visualization of segmentation results was illustrated in the supplement (Supplementary Figures 1, 2, 7–9). Quantified CT characteristics are summarized in Table 3. Survivors had smaller absolute and percentage volumes of the total pneumonia infection as compared to non-survivors (263 vs. 657 ml; 9 vs. 22%; *p* < 0.001). Similar results were observed for the GGO and consolidation regions. The average HU value for the consolidation region was lower for survivors than that for non-survivors (−62 HU vs. −51 HU; *p* < 0.001). The average HU values for the total pneumonia infection (−495 HU vs. −515; *p* = 0.62) and the GGO region (−485 HU vs. −492 HU; *p* = 0.58) did not show significant differences. The characteristics related to the pleural effusion region were similar between survivors and non-survivors.

**Table 2:** Performance of our AI system on lung field and lesion segmentation tasks evaluated on internal validation set.

**Segmentation tasks**	**Dice**
Lung field	0.97 ± 0.016
Consolidation	0.74 ± 0.21
GGO	0.81 ± 0.21
Total pneumonia infection regions	0.74 ± 0.21
Pleural effusion	0.79 ± 0.23

*GGO, ground-glass opacity; Dice, Dice Coefficient*.

**Table 3:** CT quantification indexes of 238 COVID-19 patients.

	**ALL (*n* = 238)**	**Survivor (*n* = 126)**	**Non-survivor (*n* = 112)**	***p*-value**
**Total pneumonia infection**				
Volume of total pneumonia infection (ml)	438 (142–1,125)	263 (68–746)	658 (307–1,410)	< 0.001
Ratio of total pneumonia infection (%)	15.9% (3.96–42.2%)	9.1% (1.6–37.2%)	21.8% (9.03–50.1%)	< 0.001
HU of total pneumonia infection	−501 (−571–420)	−495 (−560–434)	−515 (−573–408)	0.62
**GGO**				
Volume of GGO (ml)	220 (77–605)	156 (38–459)	336 (150–809)	< 0.001
Ratio of GGO (%)	8.1% (2.1–23.7%)	4.95% (1.02–20.5%)	11.4% (4.3–27.1%)	< 0.001
HU of GGO	−486 (−514–464)	−485 (−514–463)	−492 (−518–464)	0.58
**Consolidation**				
Volume of consolidation(ml)	61 (18–161)	43 (9–134)	96 (30–211)	< 0.001
Ratio of consolidation (%)	2.1% (0.5–6.9%)	1.3% (0.3–5.6%)	2.8% (0.8–7.5%)	0.004
HU of consolidation	−55 (−72–44)	−62 (−74–50)	−51 (−65–39)	< 0.001
**Pleural effusion**				
Volume of pleural effusion (ml)	0.0 (0.0–0.0)	0.0 (0.0–0.0)	0.0 (0.0–0.0)	0.04
Ratio of pleural effusion (%)	0.0 (0.0–0.0)	0.0 (0.0–0.0)	0.0 (0.0–0.0)	0.04
HU of pleural effusion	8.98 (4.6–23.1)	4.3 (2.1–5.1)	20.9 (7.3–24.7)	0.04
Volume of pleural effusion^*^ (ml)	13.6 (96.95)	6.9 (52.9)	21.2 (129.7)	0.04

*Data are median (IQR), n (%), or n/N (%). p-values were calculated by Mann-Whitney U-test, Chi-square test, or Fisher's exact test, as appropriate. GGO, ground-glass opacity. Since the number of patients with pleural effusion were too small, both median and IQR of pleural effusion volume were 0.00. In order to better explore the association between pleural effusion and patients with COVID-19, we also showed the mean value and standard deviation of pleural effusion volume in the row “Volume of pleural effusion*

* *(ml)”*.

Our new proposed radiologic marker, the V-HU score, was a strong univariable predictor of mortality. The score (0, 1, or 2) classified patients with COVID-19 pneumonia into three categories with respect to the risk of death: low risk; intermediate risk (HR for the comparison with low risk, 2.54; 95% CI 1.44–4.49); and high risk (HR for the comparison with low risk, 4.90; 95% CI 2.78–8.64) (Figure 2). From the Kaplan-Meier curve, the three groups have different survival probabilities (*p* < 0.001), which confirmed the high prognostic value of this radiologic biomarker. Moreover, age, sex, cerebrovascular disease, white blood cell count, neutrophil count, c-reactive protein, blood oxygen, lactic dehydrogenase, d-dimer, absolute and percentage volumes of the total pneumonia infection, GGO, consolidation, and average HU of consolidation and pleural effusion were also associated with death (see univariable analysis in Table 4).

**Figure 2:** Kaplan-Meier estimates of survival probability as a function of the number of patients at risk segregated by the V-HU score. As some patients in the intermediate-risk and the high-risk group died on the day of their first CT examination, their curves did not start from 1.0.

**Table 4:** Results from univariable cox proportional hazards regression in 238 patients with COVID-19.

	**Hazard ratio (95% CI)**	***p*-value**
**Demographics and clinical characteristics**		
Age ≥65 years	3.36 (2.22–5.07)	<0.001
Sex Men	1.84 (1.23–2.75)	0.003
Temperature ≥37.9°C	0.74 (0.51–1.07)	0.11
Comorbidity present Cerebrovascular disease	2.29 (1.36–3.85)	0.002
Comorbidity present Cardiovascular disease	1.41 (0.91–2.21)	0.13
Comorbidity present Diabetes	1.37 (0.88–2.13)	0.17
Comorbidity present Hypertension	1.43 (0.98–2.07)	0.06
**Outpatient laboratory parameters**		
White blood cell count ≥5.9 × 10^9^per L	2.46 (1.67–3.64)	<0.001
Neutrophil count ≥4.5 × 10^9^per L	2.66 (1.80–3.94)	<0.001
Lymphocyte count ≥0.8 × 10^9^per L	0.70 (0.48–1.02)	0.06
C-Reactive protein ≥3.8 mg/L	1.88 (1.29–2.74)	0.001
**Inpatient laboratory parameters**		
Blood oxygen ≥60.0	0.54 (0.37–0.79)	0.001
D-dimer ≥2.2 μg/L	1.75 (1.20–2.55)	0.004
Lactic dehydrogenase ≥316.0 U/L	2.30 (1.58–3.37)	<0.001
**Radiologic parameters**		
volume of total pneumonia infection ≥437.7 ml	2.81 (1.89–4.17)	<0.001
HU of total pneumonia infection ≥-501.1	0.88 (0.61–1.28)	0.50
Ratio of total pneumonia infection ≥15.9%	2.26 (1.54–3.32)	<0.001
volume of GGO ≥219.6 ml	2.26 (1.54–3.32)	<0.001
HU of GGO ≥-486.1	0.75 (0.52–1.09)	0.14
ratio of GGO ≥8.1%	2.25 (1.53–3.32)	<0.001
volume of consolidation ≥61.1 ml	2.18 (1.48–3.19)	<0.001
HU of consolidation ≥-55.5	2.05 (1.40–3.01)	<0.001
ratio of consolidation ≥2.1%	1.70 (1.17– 2.47)	0.01
volume of pleural effusion ≥0.0 ml	1.93 (1.03–3.60)	0.04
HU of pleural effusion ≥8.98	7.42 (1.52–36.11)	0.01
ratio of pleural effusion ≥0.0 %	1.93 (1.03–3.60)	0.04
V-HU		
0.0	1 (ref)	
1.0	2.54 (1.44–4.49)	<0.001
2.0	4.90 (2.78–8.64)	<0.001

*The V-HU score was our new proposed CT biomarker, which took both the volume of total pneumonia infection and the average HU value of consolidation into account. The V-HU score was “0” (categorized into low-risk group) if both the volume of total pneumonia infection and the average HU value of the consolidation region were less than the corresponding median values in study participants. Similarly, the V-HU score was “2” (categorized into high-risk group) only if both the volume of total pneumonia infection and the average HU value of the consolidation region were more than the corresponding median values in study participants. Other conditions were assigned to the value of “1” (categorized into intermediate-risk group). CI, confidence interval*.

Table 5 shows the four multivariable Cox models for factors associated with death. In these models, older age and higher neutrophil count were associated with higher mortality. V-HU score was an independent predictor when it was included in multivariable models, i.e., HR = 2.78 (high vs. low risk; 95% CI 1.50–5.17; *p* = 0.001) in model 1 and HR = 2.95 (high vs. low risk; 95% CI 1.59–5.47; *p* < 0.001) in model 4. Compared to outpatient care of model 2, adding the radiologic V-HU score (model 4) improved the mortality prediction (c-index: 0.728 [95% CI 0.687–0.781] vs. 0.695 [95% CI 0.661–0.754]; *p* < 0.001). Furthermore, on the basis of inpatient examination parameters the addition of the V-HU score also improved the mortality prediction (c-index of model 1: 0.734 [95% CI 0.702–0.787] vs. model 3: 0.716 [95% CI 0.682–0.768]; *p* < 0.001).

**Table 5:** Results from multivariable cox proportional hazards regression in 238 patients with COVID-19.

	**Model 1**		**Model 2**		**Model 3**		**Model 4**	
	**Hazard ratio (95% CI)**	***p*-value**	**Hazard ratio (95% CI)**	***p*-value**	**Hazard ratio (95% CI)**	***p*-value**	**Hazard ratio (95% CI)**	***p*-value**
**Demographic/clinical variables**								
Age (years)								
≥65	2.59 (1.67–4.03)	<0.001	3.03 (1.97–4.68)	<0.001	2.83 (1.82–4.39)	<0.001	2.69 (1.74–4.17)	<0.001
<65	1 (ref)	.	1 (ref)	.	1 (ref)	.	1 (ref)	.
Sex								
Men	.	.	1.39 (0.91–2.11)	0.12	1.30 (0.86–1.99)	0.22	1.30 (0.85–1.97)	0.23
Women	.	.	1 (ref)	.	1 (ref)	.	1 (ref)	.
Cerebrovascular disease (vs. not present)	0.87 (0.50–1.51)	0.62	0.86 (0.50–1.48)	0.59	0.94 (0.55–1.62)	0.83	0.76 (0.44–1.32)	0.33
**Outpatient laboratory variables**								
Neutrophil count (**× ** **9**^**9**^**per L)**								
≥4.5	1.82 (1.19–2.79)	0.01	2.09 (1.37–3.18)	<0.001	1.93 (1.26–2.95)	0.002	1.93 (1.27–2.94)	<0.001
<4.5	1 (ref)	.	1 (ref)	.	1 (ref)	.	1 (ref)	.
C-Reactive protein (mg/L)								
≥3.8	1.19 (0.77–1.82)	0.43	1.45 (0.96–2.18)	0.08	1.22 (0.79–1.88)	0.37	1.32 (0.87–2.00)	0.19
≥3.8	1 (ref)	.	1 (ref)	.	1 (ref)	.	1 (ref)	.
**Inpatient laboratory parameters**								
Blood oxygen								
≥60.0	0.81 (0.54–1.20)	0.29	.	.	0.81 (0.55–1.21)	0.31	.	.
<60.0	1 (ref)	.	.	.	1 (ref)	.	.	.
Lactic dehydrogenase								
≥316.0	1.52 (0.93–2.50)	0.09	.	.	1.66 (1.01–2.71)	0.04	.	.
<316.0	1 (ref)	.	.	.	1 (ref)	.	.	.
**Radiologic variables**								
V-HU								
0.0	1 (ref)	.	.	.	.	.	1 (ref)	.
1.0	1.62 (0.90–2.92)	0.11	.	.	.	.	1.64 (0.91–2.96)	0.10
2.0	2.78 (1.50–5.17)	0.001	.	.	.	.	2.95 (1.59–5.47)	<0.001
C-index	0.734 (0.702–0.787)	.	0.695 (0.661–0.754)	.	0.716 (0.682–0.768)	.	0.728 (0.687–0.781)	.

*CI, confidence interval; ref, reference*.

The V-HU score was also a significant predictor of death in older patients (age ≥ 65 years; for high vs. low risk, HR 3.56, 95% CI 1.64–7.71; *p* < 0.001) and younger patients (age <65 years; for high vs. low risk, HR 4.60, 95% CI 1.92–10.99; *p* < 0.001) subgroups (Figure 3). In the older patient group, both high and intermediate-risk patients characterized by the V-HU score presented poor prognosis with much lower survival rates than low-risk patients. In the younger patient group, high-risk patients still correlated with high COVID-19 mortality.

**Figure 3:** Kaplan-Meier estimates of survival probability of patients in ≥65 years group **(A)** and <65 years group **(B)** with COVID-19 as a function of the number of patients at risk segregated by V-HU score. As some patients in the intermediate-risk and the high-risk group died on the day of their first CT examination, their curves did not start from 1.0.

In addition, ablation studies were also conducted to isolate the prognostic effect of V, HU, and to compare using one integrated V-HU score against using two factors V and HU. Results were illustrated in Supplementary Table 3. The multivariable Cox model 1 which incorporate V-HU score showed a superior prognostic ability over that incorporated single V or HU and even both V and HU.

## Discussion

In this retrospective study of confirmed COVID-19 patients, we identified that the increased mortality was independently associated with the following factors: (1) older age, (2) neutrophil count over 4.5 × 10^9^/L, and (3) higher V-HU score, a new radiologic biomarker integrating both the volume of pneumonia infections and attenuation of consolidation calculated from CT images. The V-HU score can further stratify the risk in both younger (age < 65 years) and older (age ≥ 65 years) patients. Notably, the proposed V-HU score can be automatically computed by an adequately-evaluated AI-based pulmonary analysis system (18) and may produce fast, reliable, and reproducible prognostic measurement and evaluation in patients with COVID-19.

Previous studies have identified the volumes of different pneumonia infections as risk factors of patients with COVID-19 progressing to critical illness (14) or ICU admission/death (15). This study confirmed the correlation of increased infection volumes (total pneumonia infection, GGO, consolidation) and death in patients with COVID-19 in the univariable analysis. Moreover, we identified the importance of the CT attenuation in pneumonia infection regions, particularly consolidation, and introduced a new comprehensive radiologic biomarker, V-HU score, that integrating both the attenuation and volume of the pneumonia infections calculated from CT scans. The V-HU score is a strong prognostic factor of COVID-19 mortality in the univariable analysis and remained significant in the multivariable analysis. The histopathologic analysis of deceased patients with COVID-19 shows as the attenuation and volume of pneumonia infection increase, it is more likely to reduce patients' ventilation/blood flow ratio to less than the critical point. Then, insufficient oxygen between the alveoli and the pulmonary capillaries will result in the body's hypoxia and, thus, an increase in mortality (21).

In this study, patients with older age, as confirmed in univariable and multivariable analyses, had an increased risk of death. This is consistent with previous findings (10–12). The increased incidence of mortality in elderly patients could be counted for the marked decline in cell-mediated immune function and humoral immune function with aging (22). In addition, we also demonstrate that neutrophil count is a prognostic indicator of patients with COVID-19. As part of the first line of the innate immune defense, neutrophils were critical in the immunopathology of COVID-19. Continuous infiltration of neutrophils at the site of infection produces exaggerated cytokines and chemokines that might result in the “cytokine storm” and contribute to poor prognosis during COVID-19 (23). Other clinical and laboratory factors have also been shown to predict COVID-19 mortality or critical outcomes in previous studies, such as d-dimer (10), lactate dehydrogenase (15), blood oxygen saturation, C-reactive protein (14), and cardiovascular or cerebrovascular comorbidity (12). However, these factors were not independently associated with death risk in our multivariable models, though lactate dehydrogenase showed prognostic value when this radiologic factor was not included.

Our fully automated AI-based pulmonary analysis system can provide the V-HU score within 15 s per CT scan on average, greatly shortening patients' waiting time and reducing radiologists' burden in the current COVID-19 pandemic. Moreover, in situations that medical personnel and supplies are limited, such as emergency rooms, this CT-based V-HU score together with just patient age (or additionally easily accessed clinical factor, i.e., neutrophil count) can be used to quickly analyze the prognostic risk without further extra laboratory examinations reducing the burden for medical personnel.

Our study has several limitations. Firstly, this is a single-center study using retrospective data from Wuhan Central Hospital. It is unclear whether the strength of the association between the proposed radiologic marker and COVID-19 death differs in its prognostic implication across different populations. Second, not all patients had complete laboratory examinations leading to a certain number of missing variables. Although we applied an interpolation approach that took all aspects of uncertainty in the imputations into account, this may still affect the role of some factors. Thirdly, patients enrolled during the early period of the pandemic faced the shortage of medical resources. The lack of timely antivirals, and inadequate treatment might also contribute to the poor prognosis in some patients. Last but not least, in view of the absence of follow-up records for many mildly-ill patients, we did not include these patients in our analysis, which to some extent, might lead to a higher mortality rate reported in this study.

To our best knowledge, we conduct an imaging-based retrospective prognosis study of the COVID-19 mortality using a large number of non-survivors. We propose a CT-based radiologic imaging biomarker, V-HU score, integrating the volume and attenuation of the infected lung regions, and showing that it is an independent and strong predictor of death in patients with COVID-19. The V-HU score can be automatically and reliably computed from CT images by the AI algorithm. When combining it with age and neutrophil count, good prognostic performance has been achieved.

## Data Availability Statement

The original contributions presented in the study are included in the article/Supplementary Material, further inquiries can be directed to the corresponding author/s.

## Ethics Statement

The studies involving human participants were reviewed and approved by the Research Ethics Commission of Wuhan Central Hospital. Written informed consent for participation was not required for this study in accordance with the national legislation and the institutional requirements.

## Author Contributions

LYH, FA, XW, XL, ZC, LY, and LZ had the idea for and designed the study. FA, XW, XL, and ZC had full access to all of the data in the study and are responsible for the integrity of the data. LYH, FA, XW, XL, ZC, LY, and LZ take responsibility for the accuracy of the data analysis. LXG, XHL, NNL, LY, and LYH designed the AI system for CT image characteristics quantification in this study. NNL, LZ, DKJ, and LY drafted the paper. XHL, BLL, LY, LZ, JWY, DZG, and NNL did the statistical analysis. FA, XW, XL, ZC, LL, and JX interpreted the findings and analyses. All authors critically revised the manuscript for important intellectual content and gave final approval for the version to be published. HZ, ZC, XL, BLL, and LYH collected the data. LY and XHL further validated the experiments during the manuscript revision process. NNL, LY, LZ, and BLL revised the manuscript during the manuscript revision process. All authors agree to be accountable for all aspects of the work in ensuring that questions related to the accuracy or integrity of any part of the work are appropriately investigated and resolved.

## Conflict of Interest

LZ, DJ, JY, DG, and LL were employed by company PAII Inc. The remaining authors declare that the research was conducted in the absence of any commercial or financial relationships that could be construed as a potential conflict of interest.

## Abbreviations

AI: artificial intelligence
CI: confidence interval
C-index: concordance index
COVID-19: coronavirus disease 2019
CT: computed tomography
GGO: ground-glass opacity
HU: Hounsfield unit
IQR: interquartile range
V-HU: the volume of total pneumonia infection and the average Hounsfield unit (HU) of consolidation areas
HR: hazard ratio.
